The article "Survey on Mental Health Status and Quality of Life and Correlation among Patients with Permanent Stoma of Colorectal Tumor" was published in 2022. Journal: Comput Math Methods Med.

# Survey on Mental Health Status and Quality of Life and Correlation among Patients with Permanent Stoma of Colorectal Tumor

**DOI:** 10.1155/2022/5792312

**Published:** 2022-09-05

**Authors:** Yanlei Zou, Qiu Yang, Bi Guan, Xiaoyu Fu, Jia Wang, Yan Li

**Affiliations:** ^1^Department of General Surgery, Chengdu Fifth People's Hospital, Chengdu, Sichuan 611130, China; ^2^Center for Medical Research and Translation, Chengdu Fifth People's Hospital, Chengdu, Sichuan 611130, China; ^3^Nursing Department, Chengdu Fifth People's Hospital, Chengdu, Sichuan 611130, China

## Abstract

**Background:**

Colorectal cancer is one of the malignant tumors of the digestive system relatively hidden onset with unobvious early clinical symptoms. Most patients have developed into middle and late stages when they were diagnosed, missing the best period of operation. Advanced colorectal cancer has strong diffusion and metastasis with short survival time, which seriously threatens the life safety of patients.

**Objective:**

To investigate the mental health status and quality of life and the relationship between them in patients with permanent stoma of colorectal cancer.

**Methods:**

In this study, a case-control study was conducted to select 80 patients (stoma group) with colorectal cancer treated by permanent stoma surgery in our hospital from January 2020 to June 2021 and 80 patients (control group) with colorectal cancer treated by sphincter-preserving surgery at the same time. The psychological health degree and quality of life of the two groups of patients were evaluated by the psychological resilience scale (CD-RISC), the positive psychological capital questionnaire (PPQ), and the cancer patient quality of life-specific scale (QOL-LC), and a linear correlation model was used to analyze the correlation of CD-RISC score, PPQ score, and QOL-LC score.

**Results:**

The total scores of tenacity, optimism, self-improvement, and resilience of the patients in the stoma group were significantly lower than those in the control one, and the difference between them was statistically significant (*P* < 0.05); the four dimensions of self-efficacy, optimism, hope, and resilience and the total score of PPQ of patients in the stoma group were significantly lower than those in the control group, and all of the differences were statistically significant (*P* < 0.05); the somatic function, psychological function, symptoms of side effects, social function, and the total QOL-LC score of patients in the stoma one were significantly lower than those in the control one, and all of the differences were statistically significant (*P* < 0.05); the total QOL-LC score of patients in the stoma group showed a significant positive correlation with PPQ score and CD-RISC score (*r* = 0.511 and *r* = 0.608, *P* < 0.01).

**Conclusion:**

The overall level of mental health and life quality of patients with permanent stoma of colorectal cancer was worse than that of patients without stoma measures, and there was a certain correlation between patients' mental health and quality of life.

## 1. Introduction

Colorectal cancer is a common clinical malignant tumor of the digestive system, among which rectal cancer is the most common one, accounting for about 50%~60%, and low rectal cancer is more common in rectal cancer [1]. According to the World Health Organization, the incidence of colorectal cancer ranks third in the incidence of malignant tumors [2]. Colorectal cancer can cause changes in stool traits, abdominal pain, diarrhea, bloody stool, and other symptoms. In severe cases, intestinal obstruction, intestinal perforation, and other complications could also occur [3]. At present, the preferred method of clinical treatment for colorectal cancer is radical surgery, which can completely remove the lesion and save the lives of patients. However, postoperative complications can seriously affect the quality of life of patients [4].

A considerable proportion of patients with colorectal cancer needs to undergo permanent colostomy, which can lead to changes in defecation pathways and decreased defecation control ability. Improper care may also cause complications such as enterostomy infection, local dermatitis, stoma stenosis, and anastomotic fistula, which can lead to a serious decrease in the quality of life of patients. Patients are prone to anxiety, depression, inferiority, and other negative emotions, which adversely affects their mental health and leads to a decrease in treatment compliance, so as to affect their return to society [5, 6]. This study investigated the mental health status and quality of life and the relationship between them in patients with permanent colostomy of colorectal cancer.

Core tips: in this study, psychological resilience scale (CD-RISC) and positive psychological capital questionnaire (PPQ) were used to evaluate the psychological state of patients, and the quality of life of patients with colorectal cancer was evaluated by quality of life-specific scale (QOL-LC). It was found that colorectal cancer patients undergoing colostomy can have adverse effects on mental health and quality of life. This study also analyzed the relationship between them and found that the QOL-LC scores of stoma patients were positively correlated with PPQ scores and CD-RISC scores.

## 2. Materials and Methods

### 2.1. General Information

In this study, a case-control study was conducted to select 80 patients with colorectal cancer (stoma group) treated by permanent colostomy in our hospital from January 2020 to June 2021 and 80 patients with colorectal cancer (control group) treated by sphincter-preserving surgery in the same period. For the selection of research subjects, a table of random number was used.

Inclusion criteria: (1) patients were from 18 to 79 years old; (2) the diagnosis of colorectal cancer patients was based on postsurgical pathological examination results; (3) all patients underwent surgery in our hospital; (4) patients were with normal hearing, speaking, and comprehension abilities; (5) the research scheme met the basic requirements of Medical Ethics for Human Experimentation and Medical Ethics, and the informed consent was signed with the patient and his family before the operation.

Exclusion criteria: (1) combination of cancer in other sites, (2) combination of major diseases in other sites that affect the quality of survival, (3) history of mental illness, and (4) previous history of cranial surgery.

### 2.2. Scale Measurement

Resilience scale (CD-RISC) [7] consists of 25 questionnaire items and 3 questionnaire dimensions, which are assessed in terms of the patient's resilience, optimism, and self-improvement, respectively, and each questionnaire item is rated on a 5-point scale ranging from “never” to “almost always,” with a rating range of 0 to 4. With a total score of 100, the higher the score the better the patient's resilience level.

The positive psychological capital questionnaire (PPQ) [8] was compiled by Professor Zhang Kuo of Tianjin Nankai University in 2009. The scale contained 26 questionnaire items and 4 survey dimensions. The scale was scored from the four dimensions of patients' self-efficacy, optimism, hope, and resilience on a 7-point Likert scale, with a total scale score range of 26 to 182, and the scores are positively correlated with the psychological capital level of patients.

The quality of life-specific scale for cancer patients (QOL-LC) [9] was compiled by Wan Chonghua and other experts, which consists of four dimensions: physical function (six questionnaire items), psychological function (six questionnaire items), symptoms and side effects (five questionnaire items), and social function (five questionnaire items), with a total score of 220 and a significant positive correlation between the scores and the life quality of patients.

All patients were investigated by CD-RISC, PPQ, and QOL-LC and other three scales, which were completed independently by patients within a specified time frame, with a 100% recall rate. The scales were scored by two caregivers and the average values of the two results were taken.

### 2.3. Statistical Processing

Statistical software SPSS 21.0 was used for data statistics. The measurement indexes such as resilience, optimism, self-improvement, and total psychological resilience scores collected from the two groups in this study were tested by normal distribution, which were in line with approximate normal distribution or normal distribution, expressed as ($\bar{x}\pm s$). The *t*-test was used for comparison between the two groups; the *χ*^2^ test was used for comparison between groups for nonhierarchical count data such as adjuvant chemotherapy, health insurance mode, and tumor site; the relationship between life quality and PPQ score and CD-RISC score was studied by Pearson linear correlation analysis; the test level was *α* = 0.05.

## 3. Results

### 3.1. Comparison of Baseline Data between the Two Groups of Patients

There was no significant difference in age, gender, BMI, years of education, adjuvant chemotherapy, medical insurance, and tumor location between the two groups (*P* > 0.05) (Table 1).

### 3.2. Comparison of Resilience Scores between the Two Groups

The total scores of tenacity, optimism, self-improvement, and resilience of the patients in the stoma group were significantly lower than those in the control group, and the difference between them was statistically significant (*P* < 0.05) (Table 2).

### 3.3. Comparison of PPQ Scores between the Two Groups

The four dimensions of self-efficacy, optimism, hope, and resilience and the total score of PPQ of patients in the stoma group were significantly lower than those in the control group, and all of the differences were statistically significant (*P* < 0.05) (Table 3).

### 3.4. Comparison of Quality of Life Scores between the Two Groups

The somatic function, psychological function, symptoms of side effects, social function, and the total QOL-LC score of patients in the stoma group were significantly lower than those in the control group, and all of the differences were statistically significant (*P* < 0.05) (Table 4).

### 3.5. Correlation of Quality of Life with PPQ Score and CD-RISC Score

Simple linear correlation analysis showed that the total score of QOL-LC was positively correlated with PPQ score (*r* = 0.511, *P* < 0.01) and CD-RISC score (*r* = 0.608, *P* < 0.01) (Figures 1 and 2).

## 4. Discussion

Epidemiological survey found that the incidence of colorectal cancer in China was 13.29 : 100 000. Although this ratio was lower than that in Western European and American countries, the total number of colorectal cancer cases is still considerable due to the large population base in China [10–12]. In recent years, the incidence rate of colorectal cancer has shown a gradual increasing trend with the improvement of the living standard [13]. Surgery is the cornerstone of various treatments for colorectal cancer, but the surgical trauma is large, and patients suffer great physical and mental pain during perioperative period [14–16]. Although the current implementation of neoadjuvant therapy has reduced the recurrence rate of local lesions and increased the possibility of anus preservation, a considerable number of patients still have local recurrence due to the particularity of the physiological and anatomical location of the colorectal part and the lymphatic drainage pathway [17, 18].

Enterostomy, also known as artificial anus, is a section of intestinal opening artificially flipped and sewn to the abdominal wall incision after resection of the intestinal lesion to replace the function of the anus in order to solve the defecation problem of colorectal cancer patients [19, 20]. However, enterostomy causes great inconvenience to patients' life, resulting in great physical and psychological pain, and even affects their compliance with subsequent treatment [21]. CD-RISC scale is a tool to evaluate the resilience of patients. Hope and optimism represent positive attitudes towards life and the hope for rehabilitation and future life. Resilience refers to the confidence to deal with difficulties, not easily abandoned, go away from the plight and negative state as soon as possible [22, 23]. *Q* scale is the basis for evaluating the psychological capital level of patients, including four dimensions of self-efficacy, optimism, hope, and resilience [24, 25]. This study found that the total scores of resilience, optimism, self-improvement, and psychological resilience as well as the four dimensions of self-efficacy, optimism, hope, and resilience and the total score of PPQ were significantly lower in patients with stoma than in patients without stoma, which was due to the fact that colorectal cancer disease itself and the pain caused by treatment could lead to great psychological stress, and patients often had negative psychological emotions due to concerns about their condition, prognosis, and treatment costs [26, 27]. Stomatostomy has changed the normal defecation pathway, which may lead to problems such as decreased defecation control ability, odor, and infection, thereby reducing psychological resilience and self-efficacy, and unable to get out of the dilemma quickly [28, 29].

One of the current treatment goals for malignant tumors is to improve the survival quality of patients, and the QOL-LC is a common tool for evaluating the survival quality of patients with good reliability and validity. The scale can comprehensively reflect the survival quality of patients from four dimensions, including physical function, psychological function, symptoms of side effects, and social function [30, 31]. This study found that the physical function, psychological function, symptoms of side effects, social function, and QOL-LC scores of stoma patients were significantly lower than those of nonstoma patients, which suggested that the overall survival quality of patients with colorectal cancer undergoing permanent colostomy was worse than that of patients without colostomy. This is due to the change in the defecation mode of patients with enterostomy, the loss of the control function of the sphincter, and the failure to control the excretion behavior. It is necessary to wear the stoma bag for life to collect the excreta, which not only changes the body shape but also produces odors and sounds. Patients are afraid of being found and abandoned, which has a negative impact on the daily life and social activities of patients [32, 33].

The simple linear correlation analysis was also used in this study. The QOL-LC total score of colostomy patients was significantly positively correlated with PPQ score and CD-RISC score. This result suggested that there was a certain correlation between the mental health status and life quality of colorectal cancer patients with permanent colostomy. Mental health is an important part of life quality. Negative emotions can affect sleep quality, cause the body to be under stress, reduce self-efficacy, and have certain adverse effects on physical function, symptoms of side effects, and social function [34, 35].

In conclusion, the overall level of mental health and life quality of patients with colorectal cancer undergoing permanent colostomy was worse than that of patients without colostomy, and there was a certain correlation between mental health and life quality of patients.

## Figures and Tables

**Figure 1:** Scatter diagram of correlation between total QOL-LC score and PPQ score.

**Figure 2:** Scatter diagram of correlation between total QOL-LC score and CD-RISC score.

**Table 1:** Comparison of baseline data between the two groups.

Group	*n*	Age (years)	Gender (%)		BMI (kg/m^2^)	Years of education (years)	Adjuvant chemotherapy (%)	Medical insurance mode (%)		Tumor site (%)	
			Male	Female				Urban workers	Urban and rural residents	Rectal cancer	Colon cancer
Stoma group	80	53.66 ± 8.03	48 (60.00)	32 (40.00)	22.77 ± 2.16	8.55 ± 2.01	70 (87.50)	32 (40.00)	48 (60.00)	64 (80.00)	16 (20.00)
Control group	80	51.70 ± 7.94	40 (50.00)	40 (50.00)	22.48 ± 1.95	8.14 ± 1.68	66 (82.50)	39 (48.75)	41 (51.25)	69 (86.25)	11 (13.75)
*t*/*χ*^2^		1.552	1.616		0.891	1.400	0.784	1.241		1.114	
*P*		0.123	0.204		0.374	0.164	0.376	0.265		0.291	

**Table 2:** Comparison of psychological elasticity scores between the two groups ($\bar{x}\pm s$, points).

Group	*n*	Tenacity	Optimistic	Self-improvement	Total score of psychological elasticity
Stoma group	80	28.48 ± 6.41	8.64 ± 2.00	19.50 ± 4.47	56.62 ± 7.05
Control group	80	32.50 ± 5.84	9.44 ± 2.15	26.03 ± 6.15	67.97 ± 8.55
*t*		−4.146	−2.437	−7.682	−9.161
*P*		0.000	0.016	0.000	0.000

**Table 3:** Comparison of PPQ scores between the two groups ($\bar{x}\pm s$, points).

Group	*n*	Self-efficacy	Optimistic	Hope	Toughness	PPQ total score
Stoma group	80	30.76 ± 5.94	30.78 ± 5.84	27.58 ± 5.20	31.01 ± 4.98	120.13 ± 11.64
Control group	80	34.66 ± 5.50	33.75 ± 4.92	33.04 ± 6.16	34.58 ± 6.03	136.03 ± 14.58
*t*		−4.309	−3.479	−6.058	−4.083	−7.623
*P*		0.000	0.001	0.000	0.000	0.000

**Table 4:** Comparison of quality of life scores between the two groups ($\bar{x}\pm s$, points).

Group	*n*	Somatic function	Psychological function	Symptomatic side effects	Social function	QOL-LC total score
Stoma group	80	36.95 ± 5.70	31.03 ± 6.02	33.51 ± 7.46	26.33 ± 5.03	127.82 ± 13.76
Control group	80	41.14 ± 6.33	35.76 ± 7.50	38.64 ± 7.92	34.28 ± 6.05	149.82 ± 15.00
*t*		−4.400	−4.399	−4.217	−9.038	−9.667
*P*		0.000	0.000	0.000	0.000	0.000

## Data Availability

The datasets used and analyzed during the current study are available from the corresponding author upon reasonable request.
